The article "Fetal Fibronectin as a Predictor of Preterm Delivery: A Nigerian Cohort Study" was published in 2022. Journal: Biomed Res Int.

# Fetal Fibronectin as a Predictor of Preterm Delivery: A Nigerian Cohort Study

**DOI:** 10.1155/2022/2442338

**Published:** 2022-09-15

**Authors:** Cyril C. Ikeoha, Chidebe C. Anikwe, Osita S. Umeononihu, Bartholomew C. Okorochukwu, Johnbosco E. Mamah, George U. Eleje, Chukwuemeka O. Ezeama, Basil I. Nwokoye, Chigozie F. Okoroafor, Ikechukwu S. Ugwoke

**Affiliations:** ^1^Department of Obstetrics & Gynaecology, Alex Ekwueme Federal University Teaching Hospital Abakaliki, P.M. B 102 Abakaliki, Ebonyi state, West Africa, Nigeria; ^2^Department of Obstetrics & Gynaecology, Nnamdi Azikiwe University Teaching Hospital Nnewi, P.M.B 5025 Nnewi, Anambra state, West Africa, Nigeria; ^3^Department of Obstetrics and Gynecology, Federal Medical Centre Owerri, P.O. Box 1010, Owerri, Imo State, Nigeria

## Abstract

**Background:**

Fetal fibronectin is a useful biomarker in the diagnosis and management of preterm labour.

**Objectives:**

To evaluate the relationship between cervical fetal fibronectin and preterm delivery and the association between cervical fetal fibronectin level and gestational age at delivery.

**Materials and Methods:**

A prospective cohort study was performed in a tertiary hospital in Nigeria, involving equal number of pregnant women with (96) and without (96) preterm labour. Fetal fibronectin assay was done using solid-phase immunogold assay. The data were analysed using IBM SPSS version 24. Descriptive and inferential statistical analyses were done. The level of significance was *p*-value <0.05.

**Results:**

Less than half (47.9%) of the women in the study group had preterm delivery while 13.09% of the women in the control group delivered preterm. Fetal fibronectin test had a sensitivity, specificity, positive predictive value and negative predictive value of 78%, 86.5%, 71.9%, and 89.0%, respectively, a positive likelihood ratio and negative likelihood ratio of 5.76(95% CI, 3.67 – 9.64) and 0.26(95% CI, 0.16 – 0.41), respectively.

**Conclusion:**

The findings in our study value of fetal fibronectin in predicting preterm delivery. Its use will support less intervention for patients with negative results.

## 1. Introduction

Preterm delivery is a leading cause of neonatal morbidity and mortality [1–3]. The rate of preterm delivery varies globally and has been estimated to accounts for 11.1% of all live births worldwide; it ranges from 5% in most developed European countries to 18% in several African countries [1]. More than 60% of all preterm deliveries occurred in the underdeveloped regions of sub- Saharan Africa and South Asia [1]. In Nigeria, the point prevalence rate of preterm delivery varies between 6.4% and 16.9% [4–7]. Preterm delivery harms the socio-psychological wellbeing of parent [8] and is associated with a myriad of negative short and long-term effects on the neonate. Administration of antenatal corticosteroids is effective in reducing some preterm delivery complications such as respiratory distress syndrome, intraventricular haemorrhage, necrotizing enterocolitis, intensive care admissions, and systemic infections [9].

Early diagnosis is paramount in reducing preterm birth and its prohibitive costs of care [10]. The biochemical assay for fetal fibronectin appears to be the most promising method of screening for preterm delivery and has been assessed in multiple studies [11].

Fetal fibronectin is a major component of the extracellular matrix of the membranes of the amniotic sac confines at the choriodecidual junction [12]. Fetal fibronectin can be distinguished from its other family members by the presence of a unique region known as the III-CS domain [13]. Scientists have developed a monoclonal antibody called FDC-6 which specifically recognizes the III-CS domain of fetal fibronectin. In 1991, Lockwood et al. demonstrated fetal fibronectin to be an effective predictor of preterm labour in pregnant women with intact membranes and preterm birth [10]. Fetal fibronectin is elevated in cervicovaginal secretion during the first 24 weeks of pregnancy but diminishes between 24 and 34 weeks in normal pregnancies [13]. Detection of fetal fibronectin in cervicovaginal secretions between 24 and 34 completed weeks gestation is reported to be associated with preterm delivery in symptomatic and asymptomatic pregnant women [14]. In 1997, Peacemeal et al. using fetal fibronectin assay determined a negative predictive value of 99.5% for delivery within 1 week and 99.2% for delivery within 2 weeks. The positive predictive value for delivery within 1 week is 62.5%. Symptomatic pregnant women with a positive fetal fibronectin test are at increased risk for delivery at or less than 7 days and preterm delivery at less than 36 completed weeks [10]. Asymptomatic pregnant women with a positive fetal fibronectin test are at increased risk for delivery at or less than 34weeks [10, 15].

A positive fetal fibronectin test enhances the ability of the clinician to predict preterm delivery either in an asymptomatic pregnant population or a population of pregnant women presenting with equivocal symptoms [16, 17]. The majority of women with a negative fetal fibronectin test result who deliver prematurely, deliver after 34 completed weeks when serious perinatal morbidity is unlikely though possible [18, 19]. In addition, women especially symptomatic patients, with negative test results may not require severe lifestyle changes like bed rest and work restrictions which can have significant social, economic, and emotional effects [20]. With the use of fetal fibronectin test, accurate identification of women who will not deliver prematurely and thus will not benefit from referral and treatment is of the utmost importance. This identification could enhance the care that is provided to women to reduce the financial costs incurred by the health system and those with positive fetal fibronectin tests that are at increased risk for early preterm delivery will be promptly transferred to a center where they can receive treatment to enhance outcome [21]. Therefore reduction of preterm delivery through the use of fetal fibronectin assay will help reduce the complications, morbidity, mortality, and cost of caring from preterm delivery. The predictive value of fetal fibronectin in predicting preterm labour has been reported in the western population by researchers but its positive and negative predictive values and relevance in African parturients are yet to be truly verified. The study, therefore, aims to provide non-existing local data on the predictive value of fetal fibronectin in the study area. This may inform prediction and preventive management for preterm labour and hence improve obstetric outcomes within the population as the preterm delivery rate (10.59%) is high in the area of study.

Many observational studies showed that combination of cervical length and fetal fibronectin assessment may improve prediction of spontaneous preterm symptoms particularly in those with cervical length of 15-30 mm [22]. In symptomatic women qualitative fetal fibronectin testing does not improve the prediction of preterm delivery within 7 days compared with qualitative fetal fibronection testing in combination with cervical length measurement in terms of reclassification from high to low 5% risk, but it adds value across the risk range [23].

## 2. Material and Methods

### 2.1. Study Design

The study was a prospective cohort study involving pregnant women who attended antenatal clinics and those admitted into the antenatal ward of AE-FUTHA. These patients are segregated into two groups based on inclusion and exclusion criteria.

### 2.2. Group 1 (Study Group)

This group was made up of pregnant women between 28 weeks 0 day and 37weeks and 6 days who had signs and symptoms of preterm labour. The signs and symptoms of preterm labour include uterine contractions occurring at least 1 palpation of 1 contraction in 10 minutes and documented cervical changes with dilatation of not more than 3 cm.

### 2.3. Group 2 (Control Group)

This was made up of pregnant women without signs and symptoms of preterm labour between 28 weeks 0day and 37weeks and 6 days gestation who were matched for age, parity, gestational age, and booking status with women having signs and symptoms of preterm labour.

### 2.4. Study Area/Setting

This research was in Abakaliki. It is the capital of Ebonyi state in South-East Nigeria. It has 13 Local Government Areas, one urban, one semi-urban with the rest being rural. It occupies a landmass of 5935km^2^ space sharing boundaries in the west with Enugu state, Cross River State in the East, Abia state in the south, and Benue state in the north. Ebonyi state has an estimated population of 2.3 million people, while Abakaliki has 198,793 people of which 96,463 are males and 102,330 are females [22]. In Abakaliki, women of the reproductive age group constitute 20% of the people, and about 75% of the entire population dwell in the rural areas with farming as their major occupation.

Alex Ekwueme Federal University Teaching Hospital, Abakaliki (AE-FUTHA) is the only tertiary health facility located in the capital city of the state and receives referrals mostly from parts of the state and also from the neighboring states of Benue, Enugu, Cross River, and Abia. The hospital has an Obstetrics and Gynaecology department manned by 28 consultants divided into 5 teams with antenatal clinics been conducted from Monday to Friday. There are 17 beds in the antenatal ward, 50 beds in the postnatal ward, 34 beds for gynaecologic patients, and 6 beds in the labour ward. The annual antenatal clinic patient load is about 4200 clients, about 3600 deliveries occur yearly, and preterm labour formed about 10.59% of the deliveries.

### 2.5. Study Population

Pregnant women included in the study were those who consented to participate with gestational age between 28 weeks 0 day and 37 weeks +6 days, cervical dilatation of 3 cm and below, intact fetal membranes, and carrying a singleton fetus. Women diagnosed with fetal membranes rupture, antepartum hemorrhage, and intrauterine fetal growth restriction were excluded. Others excluded include women with unsure dates (with no first-trimester ultrasound scan results), diabetes mellitus, pre-eclampsia, or sickle cell disease. Women with a history of sexual intercourse or vaginal lubricant use in the 24 hours preceding recruitment were excluded however if this client comes back a week later without these conditions, she qualifies for inclusion. Each patient who consented following an informed consent process was enrolled at contact with the use of an interviewer-administered proforma. Written informed consent was obtained from the participants after a brief introduction of the researcher/research assistant, a brief detail about the research, what the participants will do to assist the researcher, and what she should expect. This section assured her of her confidentiality and that both the information obtained and the test results were used only for the research work and were treated with strict confidence.

The proforma was divided into 3 sections. Section A enquired about the bio-data and socio-demographic characteristics of all participants; section B was for patients with signs and symptoms of preterm labour while section C was for information on clinical parameters and results of investigations and feto-maternal outcomes.

### 2.6. Sample Size Determination

The formula for calculating sample size in cohort studies comparing two groups was used [23].

(1) $$\begin{array}{c} N=\frac{2\left(\text{Z}\alpha +\text{Z}\beta \right)2}{\left[\left(µ1-µ2\right)/\text{o}\right]2} \end{array}$$

Z*α* = is the value of the standardized score cutting off *α*/2 proportion of each tail of a standard normal distribution (for a two-tailed hypothesis test). This will be set at 1.96.

Z*β* = is the value of the standardized score cutting off the upper *β* proportion. This will be set at 1.282 for power (1-*β*) of 0.9.

*α*2 = is the assumed common variance in the two groups. *μ*1-*μ*2 is the difference in means of the two groups. (*μ*1-*μ*2)/*α* =0.5formedium effects.

Using the formula above

(2) $$\begin{array}{c} \text{Z}\alpha =1.96\\ \text{Z}\beta =1.282\text{ for }\left[1-\beta \right]\text{ of }0.9 \end{array}$$

*μ*_1_ - *μ*_2_ =0.5 for medium effect.

(3) $$\begin{array}{c} N=\frac{2{\left[1.96+1.282\right]}^{2}}{0.5^{2}}=\frac{2{\left[3.242\right]}^{2}}{0.5^{2}}=\frac{2\times 10.510}{0.25}=84.08 \end{array}$$

Using a 10% attrition rate =8.408.

The sample size for each group is 84.08+8.408 = 92.488 approximated to =96 for each group, therefore the total sample size for the study was 192.

### 2.7. Recruitment of Subjects

The patients included were women who were diagnosed as having clinical symptoms and signs of preterm labour. Diagnosis of preterm labour was made in a woman with uterine contractions of at least 1 palpation of 1 contraction in 10 minutes and also documented cervical changes in dilatation of not more than 3 cm. Informed consent was obtained from women that met the inclusion criteria and a detailed history is obtained to determine the risk factors present in the patient, the gestational age, and presence or absence of rupture of membranes. Physical examination was done to assess for pallor, jaundice, pedal oedema then vital signs which include temperature, pulse rate, blood pressure, and respiratory rate. The abdomen was palpated for uterine contractions, fundal height, lie, presentation. The woman is placed in a dorsal position with a lower limb flexed at the hip and knee with the legs abducted, thus exposing the vulva. A sterile apron was used to cover her legs. The sterile vaginal examination was done using a sterile disposable speculum, after washing the hands and adorning a sterile glove, to assess the cervical dilatation, vaginal bleeding, abnormal vaginal discharge, and drainage of liquor. Specimen collection was done followed by digital vaginal examination was done unless contraindicated by rupture of membrane or placenta praevia. Further management is dependent on if it is threatened or established preterm labour, the gestational age, and the presence or absence of rupture of membranes. In threatened preterm labour, the cervical dilatation is less than 4 cm and in established preterm labour, the cervical dilatation is 4 cm or above. Premature rupture of membranes was ruled out by sterile speculum examination through observing for oozing of amniotic fluid from the external cervical os on the Valsalva maneuver and pooling of the amniotic fluid in the posterior blade of the Cusco's speculum. This was followed by digital examination for dilatation and effacement of the cervix. The patients were matched with a control group of pregnant women who do not have signs and symptoms of preterm labour. They were matched for age, parity, and gestational age.

### 2.8. Outcome Measures

1. Fetal fibronectin test positivity in women with signs and symptoms of preterm labour
2. Fetal fibronectin test positivity in women without signs and symptoms of preterm labour
3. The proportion of women with detectable fetal fibronectin test positivity who delivered from 28 weeks 0day to 37 weeks 6days of gestation

### 2.9. Collection of Specimen and Test Procedure

The pregnant woman was asked to lie in a dorsal position as earlier described above. Sterile gauze soaked in normal saline was used to swab the vulva from front to back. A sterile speculum without lubricant was inserted. The speculum was then opened, locked, and kept in position to expose the cervix and posterior fornix of the vagina. Sterile polyester tipped applicator was used for specimen collection. During a speculum examination, before any examination or manipulation of the cervix or the vaginal tract, the applicator tip lightly rotated across the posterior fornix of the vagina for approximately 10 seconds to absorb cervicovaginal secretions. Subsequent attempts to saturate the applicator tip may invalidate the test. The sample was then inserted into the tube containing the extraction buffer and mixed vigorously for 10 to 15 seconds and transferred to the laboratory for analysis. Before collecting the patient's sample, the tube containing the extraction buffer was removed from the package and the cap carefully removed. As much liquid as possible was removed from the applicator by rolling the tip against the inside of the tube. The applicator was disposed of in a manner consistent with handling potentially biohazardous materials. The test strip was removed from the foil pouch making sure to handle only the labeled portion of the test strip. The area indicated by the arrows was dipped into the tube containing the extraction buffer. The test strip was not further immersed in the dip area. The tube was not recapped during test strip incubation. The test strip was allowed to stand in the extraction buffer for 10 minutes. Immediately the test strip was removed and the result was read. The quick check fetal fibronectin test is a qualitative test. A negative result indicating the absence of fetal fibronectin will appear as one line. A positive result indicating the presence of fetal fibronectin will appear as two lines (indicative of fetal fibronectin levels >50 ng/ml).

### 2.10. Principle of the Test [24]

The quick check fetal fibronectin test is a solid-phase immunogold assay. Specimens obtained from the posterior fornix are placed into an extraction buffer. A test strip with immobilized mouse monoclonal anti-fetal fibronectin antibody, human fibronectin, and goat polyclonal anti-fibronectin antibody gold conjugate is then placed in the extraction buffer. The extraction buffer migrates up the test strip by wicking; the polyclonal antibody- colloidal gold conjugate becomes re-suspended and migrates with the extraction buffer. If fetal fibronectin is present in the specimen, it will bind to the anti-human fibronectin colloidal gold conjugate. This complex migrates by capillary action across a membrane containing an immobilized monoclonal antibody specific to fetal fibronectin. The fetal fibronectin/anti fibronectin gold complex then binds to the immobilized anti-fetal fibronectin antibody-producing a visible line. If fetal fibronectin is absent from the sample, no binding occurs to the immobilized anti-fetal fibronectin antibody. Residual unbound anti-human fibronectin polyclonal antibody gold migrates further across the membrane and binds to immobilized plasma fibronectin, providing an assay control. A positive specimen will result in two visible lines; a negative specimen will result in one visible line.

### 2.11. Statistical Analysis

Analysis of data was done using SPSS (Statistical Package for Social Sciences) for Windows version 24, 2018 incorporated, Chicago, IL USA.

Description of quantitative variables were given as means, standard deviations.

The description of qualitative variables were given as numbers and percentages.

A chi-square test was used to compare proportions of categorical variables.

Student t-test was used for comparing means where applicable. The means were those of mean age, length of hospital stay.

The diagnostic accuracy of qualitative cervicovaginal fetal fibronectin in predicting preterm birth was determined using sensitivity, specificity, negative predictive value (NPV), and positive predictive values (PPV).

## 3. Results

A total of 192 women were included in the final statistical analysis of the study.  Table 1, shows that the majority of the subjects had a tertiary level of education (47.9%) and (53.1%) for the cases and control groups, respectively, P =0.002. A greater proportion of the subjects were booked (83.3%) and control (96.0%), P =0.001.

Table 2 indicates that almost half (46.9%) of the cases had negative fetal fibronectin test and 86.5% of the control had negative fetal fibronectin test. Over half (53%) of the cases tested positive for fetal fibronectin while only 13.5% of the control tested positive to fetal fibronectin, P =0.001. Almost half (46.9%) of the cases had preterm delivery-21.9% at a gestational age<34weeks+6 days and 26.0% at ≥34weeks – 36weeks+6days. Only 13.09% of the control had preterm delivery with the following percentages – 1.04% at 34weeks+6 days and 12.5% at 34-36weeks+6days gestation. Majority of the subjects; 52.08% and 86.5% for the control arm delivered at term (≥37weeks gestation), P =0.41. All the subjects (100%) in the cases arm were admitted after the test, P =0.41, while none of the control was admitted after the test, P =0.001.

GA-Gestational age.

Table 3, shows that the majority of the subjects were tested at a gestational age of 30-36weeks for cases (69.8%) and control (71.9%), P =0.75. None of the subjects in the case and control cohorts had vaginal bleeding. The majority (54.2%) of the cases had 2 uterine contractions in 10 minutes while none of the control had uterine contractions, P =0.001. Over half (52.08%) of the cases had steroid administration, while no participants in the control arm received steroids, P =0.001. The majority of the cases (91.7%) received tocolytics while none of the control received tocolytics, P =0.001.

Table 4 shows that 46.9% of the cases delivered preterm babies with (21.9% and 25.0%) delivering at a gestational age of <34 weeks +6 days and 25% at ≥34 – 36 weeks +6 days gestation, 13.54% of the control arm delivered preterm babies with 1.04% delivering at a <34 weeks +6 days and 12.5% at ≥34 – 36 weeks +6 days gestation, P =0.001. The majority of the subjects stayed for ≤3days on admission with no critical medical needs, the percentages for the cases were 82.3% and 85.4% for control, P =0.13. The mean hospital stay was 2.7 ± 1.35SD for the case and 2.3 ± 1.02SD for the control.

## 4. Discussion

The overall diagnostic performance of the qualitative cervicovaginal fetal fibronectin test in symptomatic women in predicting preterm delivery is high as shown in Table 5, with a specificity of 84.31%, and sensitivity of 86.67%. The sensitivity and specificity are comparable with the results of the study by Mohammed El Shayed et al. [25], with a calculated sensitivity and specificity of 73% and 87%, respectively, where the fetal fibronectin test improved the prediction of preterm delivery; but are in contrast to the study of Kassam M et al. [26] with a reported sensitivity and specificity of 56% and 64.8%, respectively; where it did not improve the prediction of preterm delivery.

The negative predictive value of the fetal fibronectin test in symptomatic women in this study which is 87.76% agrees with the value of 85.0% reported by Farag et al. [13]. This means that most women who tested fetal fibronectin negative tend not to deliver preterm babies. The positive predictive value of 82.98% is also similar to those reported by Farag et al. [13] which is 77.8% and also 70.6% by Kassam et al. [26] which showed that fetal fibronectin is a good marker for the prediction of preterm delivery.

The relative risk of 6.77 (95% CI, 3.16 - 14.50) for the prediction of preterm labour found in the current study in symptomatic women is comparable to the relative risk of 3.87 (95% CI, 1.10 – 13.10) to predict preterm labour reported by Jun et al. [27]. This shows that the fetal fibronectin test has a high predictive value for predicting preterm delivery. This is in contrast to the relative risk of 0.72 (95% CI, 0.52 – 1.01) noted by Berghella et al. [16] which shows a low predictive value of fetal fibronectin for predicting preterm delivery.

The positive likelihood ratio (LR+) and negative likelihood ratio (LR-) of 5.53 (95% CI, 2.89 – 10.55) and 0.16 (95% CI, 0.07 – 0.34) in this study found in symptomatic women is comparable with the findings by Berghella et al. [16] who reported positive Likelihood ratio (LR+) and negative Likelihood ratio (LR-) of 2.7 (95% CI, 1.5 – 4.9) and 0.71 (95% CI, 0.55 -0.85), respectively; this implies a high overall diagnostic performance of fetal fibronectin test in the prediction of preterm delivery.

The diagnostic performance of the qualitative fetal fibronectin test in predicting preterm delivery in asymptomatic women as shown in table 5, showed sensitivity of 75.00%, specificity of 98.75%, positive predictive value of 92.31% and negative predictive value of 95.18%.

The sensitivity and specificity which indicates good performance is similar with the results of Don Santos F et al. [28] with a sensitivity of 60% and specificity of 93%, respectively. Fetal fibronectin test was predictive of preterm delivery. But the result is in contrast to the sensitivity reported in the study by Dogra K and Tanwar M [29] which showed sensitivity of 9% but specificity of 87.5% as the specificity remained high in most studies.

Mohamed EL-Sayed ML [25] reported a PPV of 41% compared to 92.31% in asymptomatic women in our study. This suggests that using our model clinicians can be more confident in the validity of a positive test result and can accurately target interventions while avoiding treatment in women who do not need it.

NPV of 95.18% is high in asymptomatic women in this study and it remains high in most study, Mohamed EL-Sayed ML et al. [25] reported NPV of 95.5% which is similar to the one reported in this study. This high NPV enables the clinicians to reassure the patient and for possible discharge from the intensive care unit.

The positive likelihood ratio (LR+) and negative likelihood ratio (LR-) of 60.00 (95% CI 8.38 – 429.45) and 0.25 (95% CI, 0.11-0.59) in asymptomatic women in this study is comparable with the findings by Don Santos F et al. [27] who reported positive likelihood ratio (LR-) of 12.01 (95% CI, 4.70-30.68) and 0.54 (95% CI, 0.30 - 0.97), respectively, this shows the high diagnostic performance of fetal fibronectin test in the prediction of preterm delivery. The relative risk of 19.15 (95% CI, 7.26 – 50.47) as shown in asymptomatic women in this study is high. This is comparable also to the high relative risk of 6.7 (95% CI, 4.9 – 9.2) noted in the study by Kiefer et al. [30]. This also shows that the fetal fibronectin test is predictive of preterm delivery.

The accuracy of 94.79% in asymptomatic women in this study is high which is comparable to the accuracy of 84% reported by Mohamed EL Sayed ML [25] in their study which shows that the fetal fibronectin test has a high accuracy predictive value for preterm delivery.

The clinical utility of the fetal fibronectin test relates to its high negative predictive value to identify women who are at low risk of preterm delivery. It may help to avoid unnecessary hospital admissions, prolonged hospital stays, transfer to tertiary units with advanced neonatal support, and the administration of tocolysis and corticosteroids [9]. This may also help the women to avoid unnecessary lifestyle modifications like bed rest, and work restrictions which can have some impact on the social, economic, and emotional effects on the women [18].

It is important to note that a negative fetal fibronectin test does not eliminate the probability of preterm delivery. Symptomatic women with a negative fetal fibronectin test should be treated [28]. If the fetal fibronectin test is positive these patients warrant close observation and consideration for additional intervention. The decision for corticosteroid administration, tocolytic therapy, and transfer to a tertiary care center (depending on the gestational age) should be made on an individual basis given all of the clinical information and resources available [9].

The negative predictive value of fetal fibronectin is similar to the results of other studies. The test results obtained using the fetal fibronectin test will enable clinicians to make decisions based on the test result. The use of this fetal fibronectin test in the routine clinical management of patients is important to allocate resources and management to suit individual patient's needs to avoid unnecessary hospital admission, lifestyle modification, and intervention.

## 5. Limitations of the Study

Our study is a hospital-based study with its own limitations and bias. The findings from the study could not be generalized to the whole obstetric population in the study area but our findings gave an insight into the usefulness of fFN in the management of preterm labour. Our sample size could be considered a limiting factor and a multicenter study is advocated to help evaluate the veracity of our findings; this will enable the pooling of a large number of women with preterm labour for evaluation. One of the major limitations of our study is our inability to do a quantitative measurement of fFN and cervical length measurement among the women we evaluated. Addition of these parameters would have added more leverage in the use of these tools in the management of w0men at risk of preterm labour.

## 6. Conclusion

The fetal fibronectin test has a high predictive value for preterm delivery in this study. The high negative predictive value for preterm delivery will help obstetricians manage patients based on test results. Management of those that test positive should be individualized and based on patient's clinical presentations and gestational age while those with the negative test should be reassured that the risk of delivery of preterm babies is low because of the high negative predictive value of the test to maximize resources and avoid unnecessary interventions.

## 7. Recommendations

It is recommended that routine bedside qualitative fetal fibronectin tests be adopted in Nigeria and sub Saharan African countries to test those at risk of preterm delivery. More awareness of the clinical utility of the test should be made known to patients and hospital medical staff to encourage its use. The test kits should be provided to the hospitals in Nigeria at a subsidized rate by the government, local communities and non-governmental organizations. The test kits should also be made available to hospitals in rural and remote areas to enable them to transfer patients at risk of preterm delivery to higher centers where they can be appropriately managed.

## Figures and Tables

**Table 1:** Sociodemographic variables of the study population.

Variables	Case (n,%)	Control (n,%)	X^2^	p-value
Age (years)			3.68	0.16
Mean age ± SD	29.1 ± 5.73	2.53 ± 1.02		
<20	3 (3.13)	—		
20-25	26 (27)	22 (22.9)		
>25	67 (69.8)	74 (77.1)		
Tribe			4.99	0.17
Ibo	89 (92.7)	95 (98.9)		
Yoruba	4 (4.2)	1 (1.04)		
Hausa	2 (2.1)	—		
Others	1 (1.04)	—		
Marital status			3.8	0.15
Married	90 (93.8)	95 (98.95)		
Single	5 (5.2)	1 (1.04)		
Separated	—	—		
Divorced	1 (1.04)	—		
Education			10.18	0.002
No formal education	7 (7.3)	—		
Primary	8 (8.3)	3 (3.2)		
Secondary	35 (36.5)	42 (43.8)		
Tertiary	46 (47.9)	51 (53.1)		
Parity			1.26	0.53
Primigravida	21 (21.9)	26 (27.1)		
Para 1-4	67 (69.8)	65 (67.7)		
≥5	8 (8.3)	5 (5.2)		
Booking			17.5	0.001
Booked	80 (83.3)	96 (100)		
Unbooked	16 (16.7)	—		
Occupation			1.96	0.74
Trading	29 (30.2)	30 (31.3)		
Civil servant	21 (21.9)	24 (25)		
Artisan	16 (16.7)	12 (12.5)		
Farming	6 (6.3)	3 (3.13)		
Housewife	24 (25)	27 (28.1)		

**Table 2:** Maternal clinical characteristics and test results.

Variable	Case (n,%)	Control (n,%)	X^2^	p-value
GA at test			0.58	0.75
>30 wks	10 (10.4)	7 (7.3)		
30-36 wks	67 (69.8)	69 (71.9)		
>36 wks	19 (19.8)	20 (20.8)		
Cervical dilatation			—	—
<3 cm	96 (100)	96 (100)		
≥3 cm	0	0		
Test result				
Negative	45 (46.9)	83 (86.5)		
Positive	51 (53.1)	13 (13.5)		
GA at delivery			30.92	0.001
<34wks+6	21 (21.9)	1 (1.04)		
34-36wks+6	25 (26.0)	12 (12.5)		
≥37wks	50 (52.08)	83 (86.5)		
History of preterm delivery			0.19	0.41
NO	85 (88.5)	83 (86.5)		
YES	11 (11.5)	13 (13.5)		
Admitted after test			192.0	0.001
No	0	96 (100)		
Yes	96 (100)	0		

**Table 3:** Maternal clinical characteristics and drugs administered.

Variable	Case (n,%)	Control (n,%)	X^2^	P-value
GA at test			0.58	0.75
>30wks	10 (10.4)	7 (7.3)		
30-36wks	67 (69.8)	69 (71.9)		
>36wks	19 (19.8)	20 (20.8)		
Vaginal bleeding				
No	96 (100)	96 (100)		
Yes	0	0		
Uterine contractions in 10 minutes			192	0.001
Nil	0	96 (100)		
1	27 (28.1)	0		
2	52 (54.2)	0		
3	15 (15.6)	0		
4	1 (1.04)	0		
5	1 (1.04)	0		
Steroid given			67.6	0.001
No	46 (47.9)	96 (100)		
Yes	50 (52.08)	0		
Tocolytic given			162.5	0.001
No	8 (8.3)	96 (100)		
Yes	88 (91.7)	0		

**Table 4:** Gestational age at delivery and maternal length of hospital stay.

Variable	Case (n,%)	Control (n,%)	X^2^	P-value
GA at delivery			30.9	0.001
<34wks 6 days	21 (21.9)	1 (1.04)		
34-36wks 6 days	24 (25)	12 (12.5)		
≥37 wks	51 (53.13)	83 (86.5)		
Hospital stay			4.1	0.13
Mean ± SD	2.7 ± 1.35	2.53 ± 1.02		
<3 days	79 (82.3)	82 (85.4)		
4-5 DAYS	13 (13.5)	14 (14.6)		
6-7 DAYS	4 (4.2)	0		

Abbreviations: GA-Gestational age.

**Table:** (a) Symptomatic (preterm labour)

fFN test	Preterm delivery	Term delivery	Total
Positive	39	8	47
Negative	6	43	49
Total	45	51	96

**(b):** 

Sensitivity	86.67% (95% CI, 73.21% -94.95%)
Specificity	84.31% (95% CI, 71.41% -92.98%)
PPV	82.98% ((95% CI, 71.86% -90.30%)
NPV	87.76% (95% CI, 77.12% -93.84%)
LR+	5.53% (95% CI, 2.89 – 10.55%)
LR-	0.16 (95% CI, 0.07 - 0.34)
RR	6.77 (95% CI, 3.16 – 14.50)
Accuracy	85.42%(95% CI, 76.74% -91.79%)

**Table:** (c) Asymptomatic

fFN test	Preterm delivery	Term delivery	Total
Positive	12	1	13
Negative	4	79	83
Total	16	80	96

**(d):** 

Sensitivity	75.00% (95% CI, 47.62% -92.73%)
Specificity	98.75% (95% CI, 93.23% -99.97%)
PPV	92.31% (95% CI, 62.64% -98.85%)
NPV	95.18% (95% CI, 89.42% -97.88%)
LR+	60.00% (95% CI, 8.38 – 429. 45%)
LR-	0.25 (95% CI, 0.11 - 0. 59)
RR	19.15 (95% CI, 7.26 – 50.47)
Accuracy	94.79 (95% CI, 88.26% -98.29%)

Overall diagnostic performance of fetal fibronectin test in symptomatic woman as shown by sensitivity, specificity and others.

## Data Availability

The [data used to support the findings of this study are available from the corresponding author upon request.

## Additional Points

*Study at a Glance*. (i) The study is a prospective cohort study among an equal number of pregnant women with (96) and without (96) preterm labour. Fetal fibronectin assay was done using solid-phase immunogold assay. The samples were collected with sterile polyester tipped applicator from the posterior fornix and sample extracted using the extraction buffer in a test tube. A test strip was inserted and allowed for 10 minutes after which it was read. (ii) The study aims to establish a local data for the adaptation of fetal fibronectin test in the management of women with preterm labour. (iii) The study shows the predictive value of fetal fibronectin test. Our findings can inform prediction and preventive management for preterm labour in the study area and therefore improve obstetrics outcomes. *Why was the study conducted?*. (a) The predictive value of fetal fibronectin in predicting preterm labour has been reported in the western population by researchers but it's positive and negative predictive values and relevance in African parturition are yet to be truly verified. (b) The study, therefore, aims to provide non-existing local data on the predictive value of fetal fibronectin in the study area. (c) This may inform prediction and preventive management for preterm labour and hence improve obstetrics outcome within the population as the preterm delivery rate of 10.59% is high in the study area. *What does the study add to what is already known?*. (a) The clinical utility of fetal fibronectin test in Nigeria is very low especially in the rural area. (b) This study shows the feasibility of its use especially in areas with very high rate of preterm delivery. (c) This will help in early and efficient management of preterm labour and for early transfer of such patients from the rural areas (primary/secondary health facility) to Tertiary hospitals for the best management. *What are the key findings?*. (a) The study shows the high diagnostic performance of fetal fibronectin test in the diagnosis of preterm labour in both symptomatic and asymptomatic paturients. (b) This is evidenced in symptomatic (preterm labour) women by the high values of the following; sensitivity, specificity, PPV, NPV and Accuracy of 86.60%,84.31%,82.90%,87.76%,85.42%, respectively. In asymptomatic women by the following high values; sensitivity, specificity, PPV, NPV, Accuracy of 75.00%, 98.75%, 92.31%, 95.18%, 94.79%, respectively. (c) This (above) shows the high ability of fetal fibronectin test to predict preterm labour in both symptomatic and asymptomatic paturients.
